The article "Network Pharmacology-Based Strategy to Investigate the Mechanisms of Cibotium barometz in Treating Osteoarthritis" was published in 2022. Journal: Evid Based Complement Alternat Med.

# Network Pharmacology-Based Strategy to Investigate the Mechanisms of *Cibotium barometz* in Treating Osteoarthritis

**DOI:** 10.1155/2022/1826299

**Published:** 2022-07-14

**Authors:** Guang-Yao Chen, Yi-Fei Wang, Xin-Bo Yu, Xiao-Yu Liu, Jia-Qi Chen, Jing Luo, Qing-Wen Tao

**Affiliations:** ^1^Beijing University of Chinese Medicine, Beijing 100029, China; ^2^Department of TCM Rheumatology, China-Japan Friendship Hospital, Beijing 100029, China; ^3^Beijing Key Lab for Immune-Mediated Inflammatory Diseases, China-Japan Friendship Hospital, Beijing 100029, China

## Abstract

*Cibotium barometz* is a representative tonifying kidney drug and is widely used for osteoarthritis (OA) in traditional Chinese medicine. However, its regulatory mechanisms in treating OA remain to be sufficiently investigated. The main chemical components of *Cibotium barometz* were screened through the TCMID database and the corresponding targets were acquired through SwissTargetPrediction. The OA-related targets were obtained from the OMIM, Genecards, Genebank, TTD, and DisGeNET databases. The prediction of key targets and pathways of *Cibotium barometz* in the treatment of OA was achieved by constructing a compounds-targets network and performing KEGG enrichment analysis. The OA model rats were established by the Hulth method and used to explore the protective effect of *Cibotium barometz* via cartilage pathological assessment. In vitro models of OA were built by the proinflammatory factor interleukin-1*β* (IL-1*β*) induced SW1353 cells and used to validate the mechanisms predicted by network pharmacology. Network pharmacology results suggested that the therapeutic effects of *Cibotium barometz* were closely related to matrix metalloproteinase (MMP)-1, 3, 13 and inflammation-related gene COX2, which are regulated by the NF*κ*B pathway. In vivo experiments revealed that *Cibotium barometz* could effectively restrain cartilage from degeneration and inhibit the mRNA expression of MMP-1, MMP-3, MMP-13, and COX2 in cartilage. In vitro experiments indicated that *Cibotium barometz* water extract (CBWE) could significantly inhibit the expression of MMP-1, MMP-3, MMP-13, and PGE_2_ in IL-1*β*-induced SW1353 cells and markedly prevent the translocation of NF*κ*B p65 from the cytoplasm to the nuclei and decrease its phosphorylation level. After small-interfering RNA (siRNA) was used to suppress the synthesis of NF*κ*B p65 to block NF*κ*B signaling pathway, the ability of CBWE to inhibit MMP-1, MMP-3, MMP-13, and PGE_2_ was greatly reduced. *Cibotium barometz* has a chondroprotective effect on OA by inhibiting the response to inflammation and substrate degradation, and the related mechanism is associated with the inhibition of the NF*κ*B pathway.

The article "Network Pharmacology-Based Strategy to Investigate the Mechanisms of Cibotium barometz in Treating Osteoarthritis" was published in 2022. Journal: Evid Based Complement Alternat Med.

## 1. Introduction

Osteoarthritis (OA) is a degenerative joint disease characterized by joint low-grade inflammation and cartilage degradation, which is a leading contributor of the disability of the elderly [1, 2]. OA is closely related to age, obesity, and joint trauma, and has become a major public health issue worldwide with the increase in ageing and obese populations [3, 4]. In the treatment of osteoarthritis, nonsteroidal anti-inflammatory drugs (NSAIDs) can inhibit cyclooxygenase (COX) enzymes, thus exerting anti-inflammatory and pain-relieving effects [5]. However, long-term use of NSAIDs usually causes severe gastrointestinal side effects, especially in the elderly people [6]. Glucosamine sulfate (GS) and chondroitin sulfate (CS) are widely marketed as cartilage-protective supplements with good safety profiles. However, their clinical effects are still controversial [7].

In recent years, the development of drugs for disease-modifying OA drugs (DMOADs) has become a research hotspot due to the huge demand. And the main hot research directions include delaying cartilage degeneration, reducing inflammatory response, and reducing pain by blocking nerve signaling pathways [8–10]. However, the research and development of these new drugs for OA has mostly stalled in the phase III of clinical stage, and no new drugs have been approved for the treatment of OA in the past 10 years [11]. For example, tanezumab was once considered a potential drug for pain relief in OA and then rejected by the FDA and the European Medicines Agency due to safety concerns [12–14]. Effective and safe disease-modifying anti-OA drugs are still waiting to be developed. Finding potential active ingredients from natural compounds with biological activities and easy to modify is a new strategy for OA treatment. Therefore, further research on herbal medicine may contribute to the development of new drugs [15].

Traditional Chinese medicine (TCM) has a long history of treating OA, including herbs, acupuncture, and massage. Their effectiveness has been validated by a series of randomized controlled trial studies [16, 17]. In the theory of TCM, OA is closely related to “kidney deficiency,” and thus tonifying kidney drugs are often used against OA. *Cibotium barometz* is the rhizome of *Cibotium barometz* (L.) J.Smis and is referred to as a representative tonifying kidney drug. It is a key component of the prescriptions for the treatment of OA such as Duhuojisheng Tang and Gubitong Recipe [17, 18]. Meanwhile, some studies have shown that some key components of *Cibotium barometz* can promote the proliferation of chondrocytes and play a chondroprotective role [19]. Whereas the regulatory mechanisms of *Cibotium barometz* against OA remain to be sufficiently investigated, a clear understanding of which may be helpful in food supplement development against OA.

The article "Network Pharmacology-Based Strategy to Investigate the Mechanisms of Cibotium barometz in Treating Osteoarthritis" was published in 2022. Journal: Evid Based Complement Alternat Med.

Network pharmacology is a widely used technology based on systems biology for identifying biological networks and exploring their vital active ingredients and potential therapeutic targets. In recent years, network pharmacology has emerged and become increasingly popular in the field of TCM research [20–22]. Through network pharmacology, researchers have revealed the mechanism of traditional Chinese medicine in the treatment of a series of rheumatic diseases such as rheumatoid arthritis, systemic lupus erythematosus, and osteoarthritis [23–25]. This study aimed to investigate the potential mechanisms of *Cibotium barometz* in the treatment of OA by network pharmacology and verify them through in vitro and in vivo experiments.

## 2. Materials and Methods

### 2.1. Network Pharmacology Prediction

#### 2.1.1. Main Components and Related Targets Screening

The main chemical compounds of the *Cibotium barometz* were acquired from the traditional Chinese medicine integrated database (TCMID) [26]^.^ The molecular formulae of the compounds were retrieved from the PubChem database [27] and then imported into the SwissTargetPrediction database [28] for target prediction. The OA-related genes were collected from GeneCards [29], online mendelian inheritance in man (OMIM) [30], GeneBank, therapeutic target database (TTD) [31] and DisGeNET databases [32] using the keyword “osteoarthritis.” The data obtained from these databases will be aggregated. The candidate targets of the *Cibotium barometz* against OA were equal to the intersection of the *Cibotium barometz*-related targets and OA-related targets.

#### 2.1.2. Components-Targets Network Construction and Hub Targets Selection

The compounds-targets network was constructed by Cytoscape between the chemical compounds, the candidate targets of the *Cibotium barometz* against OA and their connections. The number of each target node is counted, and the top 10 compounds are considered to be the key components of *Cibotium barometz* for subsequent constituent identification. The top 20 candidate targets were chosen as mainly related genes and displayed as a barplot diagram. The targets closely related to OA were used for subsequent experimental verification.

#### 2.1.3. Kyoto Encyclopedia of Genes and Genomes Pathways Enrichment Analysis

The candidate targets of the *Cibotium barometz* against OA were analyzed by the metascape database (http://metascape.org/) to perform the Kyoto encyclopedia of genes and genomes (KEGG) enrichment analysis and obtain the important terms of enriched KEGG pathways to speculate on the specific mechanisms of the *Cibotium barometz* against OA. The pathways closely associated with OA were applied to the follow-up experimental validation.

The article "Network Pharmacology-Based Strategy to Investigate the Mechanisms of Cibotium barometz in Treating Osteoarthritis" was published in 2022. Journal: Evid Based Complement Alternat Med.

### 2.2. Experimental Verification

#### 2.2.1. Reagents and Antibodies

0.25% Trypsin-EDTA, penicillin-streptomycin, Leibovitz's L-15 medium, and phosphate-buffered saline (PBS) were purchased from Gibco. Human IL-1*β* was purchased from Peprotech. MTS and cDNA reverse transcription systems were purchased from Promega. Color prestained protein marker and 10% PAGE Gel Fast Preparation Kit were purchased from Epizyme. Polyvinylidene difluoride (PVDF) membranes and electrochemiluminescence (ECL) luminous fluid were purchased from Millipore. Fetal bovine serum (FBS) was purchased from ScienCell. The SYBR Green real-time PCR master mix was purchased from Toyobo. 5 × loading buffer, RIPA lysis buffer, phenylmethanesulfonyl fluoride (PMSF), bicinchonininc acid (BCA) kit, 4% paraformaldehyde, Triton X-100, Hematoxylin-Eosin Staining Kit, and Modified Safranine O-Fast Green FCF Cartilage Stain Kit were purchased from Solarbio Life Sciences. Column cartilage total RNA Purification Kit was purchased from TINADZ. The HiPure Total RNA mini kit was purchased from Magen. Fluorescent mounting medium with DAPI (4,6-diamidino-2-phenylindole) was purchased from Zhongshan Jingqiao Biotechnology. Human matrix metalloproteinase (MMP)-3 enzyme-linked immunosorbent assay (ELISA) kits (DMP300) were purchased from R&D. Human MMP-1 (KA0390) and MMP-13 (KA1600) ELISA kits were purchased from Novus Biologicals. Prostaglandin E_2_ (PGE_2_) ELISA kits (EIA-4164) were purchased from DRG. Polymerase chain reaction (PCR) primers for MMP-1, MMP-3, MMP-13, NF*κ*B p65, and NF*κ*B p65 siRNA were synthesized by Tsingke Biotechnology Co., Ltd., whose sequence is presented in Table 1.

MMP-1 antibody (10371-2-AP) was purchased from Proteintech. MMP-3 antibody (ab53015), and MMP-13 antibody (ab39012) were purchased from Abcam. NF*κ*B p65 antibody (8242T) and I*κ*B-*α* antibody (4814T) was purchased from Cell Signaling. Lamin B1 antibody (YT5180) and phospho-NF*κ*B P65 (S276) (YP0187) were purchased from Immunoway. *β*-Actin antibody (TA-09), horseradish peroxidase (HRP)-conjugated goat anti-mouse IgG (ZB-5305), HRP-conjugated goat anti-rabbit IgG (ZB-2301), and Alexa Fluor 488-conjugated Goat anti-Rabbit IgG (*H* + *L*) (ZF-0511) were purchased from Zhongshan Jingqiao Biotechnology.

#### 2.2.2. Preparation of Drugs

*Cibotium barometz* water extract (CBWE) was purchased from Shanghai Yuan Ye Bio-Technology Co., Ltd, China. The *Cibotium barometz* was processed according to the method recommended by the Chinese Pharmacopoeia. The dried root of *Cibotium barometz* (L.) J. Smith was cut into slices and mixed with sand before being stir-fried. Stir-fry was stopped when the fluff on the surface was burnt brown. The sand and the fluff were removed after cooling down. CBWE was collected based on the following protocol: the processed *Cibotium barometz* slices were cut into small pieces and 10-fold distilled water was added. Then the solution was heated up to 100°C and the kettle was kept boiling for 1 hour. The process was repeated three times, and three times the decoctions were mingled and concentrated to 60 ml. After the solution cooled down to room temperature, an equal volume of anhydrous ethanol was added and mixed thoroughly. The mixture was put in the refrigerator at 4°C for 12 h and the precipitation was removed by centrifugation. The supernatant was subjected to distillation under reduced pressure until the mixture became a density of 1.08 g·cm^−3^. The obtained solution was concentrated under vacuum, spray-dried, and then stored in a refrigerator at −20°C.

The article "Network Pharmacology-Based Strategy to Investigate the Mechanisms of Cibotium barometz in Treating Osteoarthritis" was published in 2022. Journal: Evid Based Complement Alternat Med.

#### 2.2.3. Liquid Chromatography-Mass Spectrometry

Liquid chromatography-mass spectrometry (LC-MS) was used to detect whether the key components of Cibotium Barometz predicted by network pharmacology are available in CBWE. 1 mL of deionized water was mingled with 20 mg of CBWE and sonicated for 30 min. After centrifugation (12600 g/min, 10 min), the supernatant was filtered through a microporous membrane (0.45 *μ*m pore size). The sample was then injected into a Nexera high-performance liquid chromatograph (Japan Shimadzu Co., Ltd) coupled to the SCIEX 5600 Triple-TOF mass spectrometer (Sciex, Toronto, Canada). The LC-MS results were compared with MassBank online Spectral Database (https://massbank.eu/MassBank/), The ReSpect DB (http://spectra.psc.riken.jp), and GNPS platform (https://gnps.ucsd.edu/) were employed to identify key components of CBWE.

#### 2.2.4. Animals and Modeling

18 six-week-old male SD rats were purchased from SPF (Beijing) Biotechnology Co., Ltd. and raised in the Barrier Environmental Animal Laboratory of China-Japan Friendship Hospital. All rats were housed in the same animal facility with a temperature of 21 ± 2°C, humidity of 50 ± 20%, and a 12-h light/dark cycle. Ethical approval was granted by the Animal Ethic Committee of China-Japan Friendship Hospital (No. zryhyy-21-21-05-14). After being bred for one week to adapt to the feeding environment, 18 rats were divided randomly and equally into three groups (*n* = 6/group) with the use of a random digit table: the blank control group, Hulth model group, CBWE treated group.

The article "Network Pharmacology-Based Strategy to Investigate the Mechanisms of Cibotium barometz in Treating Osteoarthritis" was published in 2022. Journal: Evid Based Complement Alternat Med.

The knee OA was established in the Hulth model group and the the CBWE treated group by the Hulth method under isoflurane anesthesia, the surgical carried out as previously described [33]. Rats in the blank control group were only anesthetized and cut the epidermis without destroying the joint structure. All the rats were administered a prophylactic antibiotic of 20000 U penicillin after the operation for 3 days to avoid infection.

#### 2.2.5. Drug Intervention and Sample Collection

The maximum clinical dosage of *Cibotium barometz* is 30 g every day. The reference body weight of an adult is 60 kg. Thus, for an adult, the dose of *Cibotium barometz* (raw herb) is 0.5 g/kg. According to the body surface area formula, the dose for rats is 6.3 times that of humans, so the dose of *Cibotium barometz* (raw herb) for rats is 3.15 g/kg. Drug intervention started 3 days after Hulth modelling and continued for 28 days. After the end of the intervention, rats were anesthetized with isoflurane, and the serum and knee joints were obtained for subsequent experiments.

#### 2.2.6. Cell Culture

The SW1353 cell line (ATCC, USA) was first separated from a primary chondrosarcoma of the right humerus of a 72-year-old Caucasian female [34]. Due to resembling chondrocytes phenotypically, SW1353 cells were often applied to exploring the mechanisms of OA [35]. The SW1353 cells were purchased from Beijing Zhongkezhijian Biotech Co., Ltd. After resuscitation, the SW1353 cells were cultured with complete Leibovitz's L-15 medium, containing 89% Leibovitz's L-15 medium, 10% FBS, and 1% Penicillin Streptomycin (Special attention should be paid to this since L-15 medium does not have an appropriate pH buffer system. In order to avoid drastic changes in the pH of the medium, cells should be cultured in a humid incubator at 37°C without additional CO_2_). The cell culture medium was replaced every 2-3 days and passaged at a ratio of 1 : 2 to 1 : 3 after the digestion of 0.25% Trypsin-EDTA.

#### 2.2.7. Cell Viability Detection

Cell viability was estimated by MTS methods and used as the basis for drug intervention concentrations. 2 × 10^4^ SW1353 cells and 100 *μ*l of complete medium were planted in a 96-well plate. After the cells adhered to the wall, CBWE solution was added in each well with final concentrations of which in each well were 100, 200, 300, 400, 500, and 600 mg/L in the presence or absence of 10 ng/mL IL-1*β*. After 12 hours of incubation, the drug-containing medium was discarded, and serum-free L-15 medium was added to incubate for another 4 hours. 20 *μ*l of MTS reagent was added, and 4 hours later, the optical density (OD) value of each well was detected at 490 nm by a microplate reader (Molecular Devices, USA). The cell viability calculation formula is as follows: viability (%) = 100 × (OD of treated sample-OD of medium)/(OD of control sample-OD of medium). The highest concentration that does not cause significant adverse effects on cell proliferation is considered the optimal intervention concentration.

The article "Network Pharmacology-Based Strategy to Investigate the Mechanisms of Cibotium barometz in Treating Osteoarthritis" was published in 2022. Journal: Evid Based Complement Alternat Med.

#### 2.2.8. Pathological Assessment of Articular Cartilage

After the knee joints were separated, cutting the femur and tibia/fibula 1 cm above and below the joint line, they were soaked and fixed with 4% neutral formalin solution for 72 h. The specimens were then immersed in a 10% EDTA solution for 8 weeks of decalcification. The femoral head was cut along the sagittal plane, rinsed with distilled water, and placed in an embedded box. Serial knee sections of exactly 5 *μ*m thickness from the middle part of the knee were obtained to prepare slides. Articular cartilage sections were stained with hematoxylin and eosin (H&E). Specifically, after staining with hematoxylin (300 sec), sections were stained with eosin solution for 30 sec.

#### 2.2.9. RNA Isolation and Real-Time PCR

Total RNA is extracted and purified by adsorption columns and collection pipes according to the manufacturer's instructions. The RNA concentration and quality were quantified using a NanoDrop spectrophotometer (Thermo Scientific, USA). 1 *μ*g total RNA, 4 *μ*g MgCl_2_, 2 *μ*l reverse transcription buffer, 2 *μ*l dNTP mixture, 0.5 *μ*l recombinant RNasin ribonuclease inhibitor, 0.63 *μ*l AMV reverse transcriptase, 1 *μ*l Oligo (dT)15 primer and nuclease-free water to a final volume of 20°ul were used to construct a transcription system (A3500, Promega, USA). The mixture was heated at 42°C for 15 min, then heated at 95°C for 5 min and cooled down to 4°C finally.

Real-time PCR was performed with SYBR Green real-time PCR master mix (QPK-201, Toyobo, Japan). A 20 *μ*l of reaction system included SYBR Green real-time PCR master mix (10 *μ*l), cDNA (2 *μ*l), gene forward, reverse primer (10 *μ*mol/L, 0.8 *μ*l), and distilled water (7.2 *μ*l). Real-time PCR was performed on a QuantStudio Real-Time PCR cycler with the following protocol: preheated at 95°C for 60 s, then heated at 95°C for 15 s, 60°C for 15 s, and 72°C for 45 s in a cycle. A total of 40 cycles were completed and finally the CT value was obtained. The relative expression was analyzed based on the 2^−△△Ct^ method using the following equations: △△Ct = (Ct gene target–Ct gene reference) treatment–(Ct gene target–Ct gene reference) control and fold change = 2^−△△Ct^.

#### 2.2.10. Western Blotting

The cells were lysed by RIPA lysate buffer (containing 1% PMSF and 1% phosphatase inhibitor) and placed on ice for 25 min. The cell lysate was further centrifuged (4°C, 10000 r/min, 5 min) to remove impurities, and the supernatant was collected. The BCA method was used to detect the concentration of each sample, and it was boiled with 5 × loading buffer. The 10% PAGE Gel Fast Preparation Kit was used to prepare the SDS-PAGE electrophoresis gel according to the manufacturer's instructions. The color prestained protein marker and the samples were added to the gel hole for electrophoresis. Gel electrophoresis was carried out at 120 V, and the proteins in the gel were transferred onto the PVDF membrane (70 V, 55 min). After blocking with 5% nonfat milk powder in TBST for 1 h, the PVDF membrane was incubated with the appropriate concentration of primary and secondary antibodies. Finally, the protein blot was obtained by using the ECL luminous fluid and chemiluminescence system (Biorad, USA) and analyzed by ImageJ software.

The article "Network Pharmacology-Based Strategy to Investigate the Mechanisms of Cibotium barometz in Treating Osteoarthritis" was published in 2022. Journal: Evid Based Complement Alternat Med.

#### 2.2.11. ELISA

The concentrations of MMP-1, MMP-3, MMP-13, and PGE_2_ were determined using a commercial ELISA kit according to the manufacturer's instructions. The OD value of standard wells and sample wells was detected at 450 nm wavelength by a microplate reader. Curve Expert 1.3 software was used to generate the standard curves and calculate the concentration of each sample.

#### 2.2.12. Immunofluorescence

After the intervention, the cells were washed twice with PBS and then fixed with 4% paraformaldehyde. 0.1% Triton X-100 was used to penetrate the cytomembrane, and the cells were blocked using 1 × animal free blocking solution for 1 h. Primary antibody was then added and incubated at 4°C overnight. After discarding the primary antibody, Alexa Fluor 488-conjugated Goat anti-Rabbit IgG (*H* + *L*) was added and incubated at room temperature for 1 h. The plate was covered with fluorescent mounting medium with DAPI (4,6-diamidino-2-phenylindole). Finally, the location of target protein and DAPI was observed by an inverted fluorescence microscope (Zeiss, Germany).

### 2.3. Statistical Analysis

SPSS 20.0 was used for statistical testing. Continuous variables are presented as the mean values ± standard deviation (SD). The statistical difference between the two groups was assessed by Student's *t*-test. *P* < 0.05 was considered as significant.

## 3. Results

### 3.1. Prevention of CBWE on the Cartilage Degradation of OA Rats

The OA model was established by the Hulth method and intervened by CBWE. A cartilage pathology assessment was performed to evaluate the condition of the knee joints of the rats in each group. The results of HE staining of the knee joint suggested that CBWE could significantly relieve cartilage degeneration in OA model rats (Figures 1(a)–1(c)). Mankin's scoring of cartilage from CBWE-treated rats implied that CBWE had an ameliorative effect on cartilage degeneration (Figure 1(d)).

The article "Network Pharmacology-Based Strategy to Investigate the Mechanisms of Cibotium barometz in Treating Osteoarthritis" was published in 2022. Journal: Evid Based Complement Alternat Med.

### 3.2. Network Pharmacology Predication of *Cibotium barometz* against OA

By searching the TCMID database, a total of 26 compounds and 399 targets of *Cibotium barometz* were obtained after removing the duplicates. A total of 3556 known OA-related targets were screened in the GeneCards database, of which 209 targets were *Cibotium barometz* against OA (Figure 2(a)). The compounds-targets-network of *Cibotium barometz* against OA is shown in Figure 2(b). The barplot of the top 10 compounds in Compounds-targets-network is shown in Figure 2(c), which is considered to be key to the treatment of OA with *Cibotium barometz*. The barplot of targets sorted by the number of nodes is shown in Figure 2(d), where the matrix metalloproteinases involved in the process of cartilage degradation, PTGS2, participate in the synthesis of PGE_2_ by regulating the COX2 enzyme, crucial for the inflammatory response of OA. Thus, MMP1, MMP3, MMP13, and COX2 are considered to be key targets in the treatment of OA in *Cibotium barometz*. The pathways of *Cibotium barometz* in the treatment of OA predicted by KEGG are shown in Figure 2(e), of which the NF*κ*B pathway is closely related to OA and verified by subsequent experiments.

### 3.3. Liquid Chromatography-Mass Spectrometry of CBWE

The top 10 compounds in the compounds-targets-network of *Cibotium barometz* against OA are considered to be the key components of *Cibotium barometz* for the treatment of OA. Liquid chromatography-mass spectrometry results showed all compounds are available in CBWE (Figure 3) and the information about these compounds is in Table 2.

### 3.4. Effect of CBWE on Matrix Metalloproteinases and COX2 In Vitro

The mRNA levels of MMP1, MMP3, MMP13, and COX2 in the cartilage of the OA model group increased, compared with the blank control group, but these changes could be reversed by CBWE (Figure 4).

### 3.5. Effect of CBWE on Cell Viability

SW1353 cells were treated with different concentrations of CBWE (100, 200, 300, 400, 500, and 600 *μ*g/mL), with or without 10 ng/mL IL-1*β*. Results showed that 100, 200, 300, 400, and 500 *μ*g/mL CBWE had no obvious effect on cell viability, whereas 600 *μ*g/mL CBWE notably suppressed the cell viability, and IL-1*β* did not show a significant effect on the viability of SW1353 cells (Figure 5). Thus, 500 *μ*g/mL was chosen as the maximum intervention concentration for CBWE. Half the maximum (250 *μ*g/mL) and a quarter of the maximum (125 *μ*g/mL) were used as medium-dose and low-dose intervention concentrations, respectively.

The article "Network Pharmacology-Based Strategy to Investigate the Mechanisms of Cibotium barometz in Treating Osteoarthritis" was published in 2022. Journal: Evid Based Complement Alternat Med.

### 3.6. Effect of CBWE on COX2 and PGE2 In Vivo

After being treated with 10 ng/ml IL-1*β*, the mRNA levels of COX2 in cell lysate and PGE_2_ secreted in media appreciably increased. CBWE can significantly inhibit the abnormal alternation of COX2 mRNA and PGE_2_ with a dose-dependent effect (Figure 6).

### 3.7. Effect of CBWE on Matrix Metalloproteinases In Vivo

After being treated with 10 ng/ml IL-1*β*, the mRNA levels, the protein levels in cell lysates and the secreted protein levels in cell culture supernatant of MMP-1, MMP-3, and MMP-13 were significantly increased. The intervention of CBWE can notably suppress the expression of MMP-1, MMP-3, and MMP-13 at the mRNA level (Figure 7), protein level in cell culture supernatant (Figure 8) and cell lysates (Figure 9), which also showed a dose-dependent effect.

### 3.8. Effect of CBWE to the NF*κ*B Pathway

After being treated with 10 ng/ml IL-1*β* 30 min, the Western blot results showed that the NF*κ*B p65 in the cell lysates displayed no significant change but the phosphorylation level of NF*κ*B p65 was significantly increased, accompanied by a significant decrease in IKB-*α*. After being pretreated with CBWE for 1 h, the level of phosphorylation of NF*κ*B p65 exhibited a significant increase and the level of IKB-*α* decreased with a dose-dependent effect (Figure 10). The immunofluorescence results suggested that NF*κ*B p65 translocated into the nuclei from the cytoplasm after being pretreated with IL-1*β*, and that a high dose of CBWE can suppress the nuclear translocation of NF*κ*B p65 to some extent (Figure 11).

### 3.9. Effect of CBWE after the Inhibition of NF*κ*B Pathway

Transfections on siRNAs of NF*κ*B P65 were performed to block the NF*κ*B pathway. On this basis, CBWE was used to intervene in SW1353 cells stimulated by IL-1*β*. Results showed that the expression of PGE_2_ and matrix metalloproteases in cell culture supernatant were significantly decreased after blocking the NF*κ*B pathway, and these indicators showed no significant change though CBWE was given (Figure 12). This indicates that the CBWE acts as a chondroprotective agent mainly through the NF*κ*B pathway.

## 4. Discussion

In the TCM theoretical system, *Cibotium barometz* has the effect of tonifying the liver and kidney, strengthening the waist and knee, and removing dampness. In the clinic, *Cibotium barometz* was applied to degenerative diseases and inflammatory arthropathies such as osteoarthritis, osteoporosis, lumbar disc herniation, rheumatic arthritis, and ankylosing spondylitis. Relevant studies have shown that active ingredients of *Cibotium barometz* have various pharmacological properties, such as antioxidant, anti-inflammatory, liver-protecting, and osteoclast-suppressive effects [19, 36–39]. This study confirmed that *Cibotium barometz* is able to ameliorate cartilage degeneration in OA rats modelled by the Hulth method, which indicates that *Cibotium barometz* has a good therapeutic effect on OA.

The article "Network Pharmacology-Based Strategy to Investigate the Mechanisms of Cibotium barometz in Treating Osteoarthritis" was published in 2022. Journal: Evid Based Complement Alternat Med.

OA used to be believed to be due to normal daily wear and tear of joints, while recent studies have illustrated that the inflammatory response occupies a crucial position in the progression of OA [11, 40]. Negative factors such as joint trauma, mechanical stimulation, and apoptosis of chondrocytes may cause inflammatory response in chondrocytes [41, 42]. NF*κ*B pathway plays a key role in the inflammatory response of chondrocytes [43, 44]. When the upstream pathway activates firstly I*κ*B kinase (IKK) and in return leads to serine phosphorylation of the I*κ*B subunit in the NF*κ*B p65-NF*κ*B p55-I*κ*B trimer, allowing the I*κ*B subunit to be ubiquitinated and then degraded by proteases, NF*κ*B p65-NF*κ*B p55 dimer is released from the cytoplasm to the nucleus. Then, NF*κ*B p65-NF*κ*B p55 dimer initiates related transcriptional processes [45].

The NF*κ*B pathway is involved in the development and progression of OA mainly through its effect on the transcription of inflammatory factors and cartilage matrix hydrolases [46]. After activation of the NF*κ*B pathway inflammatory mediators such as COX2, IL-6, and TNF-*α* are transcribed, further exacerbating the inflammatory response in the joint [47]. Concurrently, the activation of the NF*κ*B pathway in chondrocytes can entail the synthesis and release of large amounts of matrix metalloproteinases and the breakdown of the balance between synthesis and hydrolysis of cartilage ECM, which is responsible for cartilage degeneration.

According to network pharmacology, the regulatory network of *Cibotium barometz* against OA suggests that *Cibotium barometz* against OA is tightly interrelated with the regulatory genes COX2, as well as MMP-1, MMP-2, MMP-3, MMP-9, and MMP-13. COX2 regulates the synthesis of PGE_2_ through enzymatic catalysis. NASIDs drugs act as analgesics and reduce inflammation by curbing COX enzyme activity and are recommended as first-line drugs by most guidelines [48, 49]. Among matrix metalloproteinases, MMP-1, MMP-3, and MMP-13 are most closely implicated in OA. Consequently, PGE_2_, MMP-1, MMP-3, and MMP-13 were used in later experimental validation. The KEGG enrichment analysis revealed that the NF*κ*B pathway is strongly associated with the treatment of OA by *Cibotium barometz*. It is therefore reasonable to assume that the *Cibotium barometz* inhibits COX2, MMP-1, MMP-3, and MMP-13 via the NF*κ*B pathway.

The article "Network Pharmacology-Based Strategy to Investigate the Mechanisms of Cibotium barometz in Treating Osteoarthritis" was published in 2022. Journal: Evid Based Complement Alternat Med.

The experiments have proven that after stimulating SW1353 cells with 10 ng/mL IL-1*β*, the level of PGE_2_ was increased, suggesting that the inflammatory response was activated. At the same time, the expression of MMP-1, MMP-3, and MMP-13 was also increased in mRNA and protein levels. After CBWE intervention, the expression of PGE_2_ decreased, suggesting that *Cibotium barometz* can inhibit the inflammatory response of IL-1*β*-induced SW1353 chondrocytes and showed a dose-dependent effect. Western blot results suggested IL-1*β* intervention notably increased phosphorylation level of NF*κ*B p65 and NF*κ*B p65 in the nucleus, and immunofluorescence showed the translocation of NF*κ*B p65 from the cytoplasm to the nucleus, which indicated the abnormal activation of NF*κ*B pathway. CBWE can appreciably reverse the above changes with a dose-depend effect, suggesting CBWE may exert its inhibitory effect on the expression of PGE_2_, MMP-1, MMP-3, and MMP-13 through suppressing NF*κ*B pathway.

To examine the key role of NF*κ*B in the treatment of OA in *Cibotium barometz*, NF*κ*B signaling pathway was blocked by transfected siRNA of NF*κ*B p65. After that, the inhibitory effect of CBWE on PGE_2_, MMP-1, MMP-3, and MMP-13 was notably weakened, confirming that *Cibotium barometz* exerts its therapeutic effect on OA mainly through NF*κ*B signaling pathway.

In conclusion, in this study, we demonstrated that the chondroprotective effect of *Cibotium barometz* is mainly achieved through the inhibition of NF*κ*B pathway. In addition, we have identified flavonoids as key components of *Cibotium barometz* for the treatment of OA in our network pharmacology predictions, and in the future, we will purify total flavonoids from *Cibotium barometz* to provide a basis for further food supplement development for the treatment of OA.

## Figures and Tables

**Figure 1:** Effect of CBWE on cartilage degradation of OA model rats. HE staining of knee joints of each group: (a) The blank control group. (b) OA model group. (c) CBWE treated group. (d) Mankin's scoring of cartilage tissue of each group. ^*∗*^*P* < 0.05 compared with the blank control group, ^Δ^*P* < 0.05 compared with the Hulth model group.

**Figure 2:** Network pharmacology predication of *Cibotium barometz* against OA. (a) The intersection between the *Cibotium barometz*-related targets and OA-related targets. (b) The compounds-targets-network of *Cibotium barometz* against OA. (c) The barplot of the top 10 compounds in Compounds-targets-network. (d) The barplot of the top 20 targets sorted by target connectivity. (e) The pathways of *Cibotium barometz* in the treatment of OA predicted by KEGG.

The article "Network Pharmacology-Based Strategy to Investigate the Mechanisms of Cibotium barometz in Treating Osteoarthritis" was published in 2022. Journal: Evid Based Complement Alternat Med.

**Figure 3:** Identification of key components of *Cibotium barometz* by liquid chromatography-mass spectrometry.

**Figure 4:** The mRNA expression of MMP1, MMP3, MMP13, and COX2 in rat cartilage in each group. (a) The mRNA expression level of MMP1. (b) The mRNA expression level of MMP3. (c) The mRNA expression level of MMP13. (d) The mRNA expression level of COX2 in (a) the blank control group, (b) OA model group, and (c) CBWE treated group. ^*∗*^*P* < 0.05 compared with the blank control group, ^#^*P* < 0.05 compared with the Hulth model group.

**Figure 5:** The viability of SW1353 cells after treatment with different concentrations of *Cibotium barometz* water extract (CBWE) and IL-1*β* (10 ng/mL). (a) SW1353 cells were treated with different concentrations of CBWE alone for 12 h (^*∗*^*P* < 0.05: cell viability increase compared with the control group). (b) SW1353 cells were treated with different concentrations of CBWE with or without IL-1*β* (10 ng/mL) for 12 h and there were no significant differences among groups with the same CBWE concentration. The data are derived from three independent experiments and expressed as the mean ± standard deviation.

**Figure 6:** Effect of different concentration of CBWE on levels of COX2 and PGE2 in IL-1*β*-induced SW1353 cells. Cells were pretreated with 125, 250, and 500 *μ*g/mL of *Cibotium barometz* water extract (CBWE) respectively and then stimulated with 10 ng/mL IL-1*β* for 12 h. (a) COX2 expression level in cell lysate detected by Western Blot. (b) PGE_2_ expression level in media detected by ELISA. The data were derived from three independent experiments and expressed as the mean ± standard deviation. (^*∗*^*P* < 0.05 compared with the control group; ^#^*P* < 0.05 compared with the IL-1*β*-treated group).

**Figure 7:** The mRNA expression levels of MMP-1, MMP-3, and MMP-13 in IL-1*β*-induced SW1353 cells treated with CBWE. Before stimulation with 10 ng/mL IL-1*β* for 12 h cells were pretreated with 125, 250, or 500 *μ*g/mL CBWE for 1 h. The data are derived from three independent experiments and expressed as the mean ± standard deviation. (^*∗*^*P* < 0.05 compared with the control group; ^#^*P* < 0.05 compared with the IL-1*β*-treated group).

**Figure 8:** The protein levels of MMP-1, MMP-3, and MMP-13 in the supernatant detected by ELISA. Before stimulation with 10 ng/mL IL-1*β* for 12 h cells were pretreated with 125, 250, or 500 *μ*g/mL CBWE for 1 h. The data are derived from three independent experiments and expressed as the mean ± standard deviation. (^*∗*^*P* < 0.05 compared with the control group; ^#^*P* < 0.05 compared with the IL-1*β*-treated group).

The article "Network Pharmacology-Based Strategy to Investigate the Mechanisms of Cibotium barometz in Treating Osteoarthritis" was published in 2022. Journal: Evid Based Complement Alternat Med.

**Figure 9:** The protein levels of MMP-1, MMP-3, and MMP-13 measured by Western blot. Before stimulation with 10 ng/mL IL-1*β* for 12 h cells were pretreated with 125, 250, or 500 *μ*g/mL CBWE for 1 h. The data are derived from three independent experiments and expressed as the mean ± standard deviation. (^*∗*^*P* < 0.05 compared with the control group; ^#^*P* < 0.05 compared with the IL-1*β*-treated group).

**Figure 10:** Effects of CBWE on the phosphorylation level of NF*κ*B p65 and NF*κ*B p65 level in the nucleus in IL-1*β*-induced SW1353 cells. Before stimulation with 10 ng/mL IL-1*β* for 30 min, cells were pretreated with CBWE (125, 250, or 500 *μ*g/mL) for 1 h. NF*κ*B p65 and phosphorylation of NF*κ*B p65, NF*κ*B p65 in the nucleus were measured by Western blotting. Lamin B1 and *β*-actin were used as internal references for the nuclear and cytoplasmic fractions, respectively. The data are derived from three independent experiments and expressed as the mean ± standard deviation (^*∗*^*P* < 0.05 compared to the control group; ^#^*P* < 0.05 compared to the IL-1*β*-treated group).

**Figure 11:** The cells were pretreated with *Cibotium barometz* water extract (CBWE) (500 *μ*g/ml) for 1 h before IL-1*β* treatment (10 ng/ml). After 30 min of incubation, the localization of NF*κ*B p65 was visualized with fluorescence microscopy after immunofluorescence stained with anti-NF*κ*B p65 antibody (green). The cells were also stained with DAPI to visualize the nuclei (blue).

**Figure 12:** Effect of CBWE on PGE_2_ and MMPs levels after blocking NF*κ*B pathway by transfection of NF*κ*B p65 siRNA. The data are derived from three independent experiments and expressed as the mean ± standard deviation. (^*∗*^*P* < 0.05 compared to the control group; ^#^*P* < 0.05 compared to the IL-1*β*-treated group; ^Δ^*P* < 0.05 compared to the NF*κ*B P65siRNA treated group).

**Table 1:** Prime sequences for quantitative real-time PCR and siRNA.

Gene name	Sequence (5′-to-3′)
Human MMP-1 Sense	CTGTTTTCTGGCCACAACTG
Human MMP-1 Antisense	GGAAGCCAAAGGAGCTGTAG
Human MMP-3 Sense	TTGGCCATCTCTTCCTTCAG
Human MMP-3 Antisense	GAAACCTAGGGTGTGGATGC
Human MMP-13 Sense	GTGCCCTTCTTCACACAGAC
Human MMP-13 Antisense	AGAGCAGACTTTGAGTCATTGC
Human NF*κ*B p65 Sense	AGGAGCACAGATACCACCAAGACC
Human NF*κ*B p65 Antisense	AAGCAGAGCCGCACAGCATTC
Human GAPDH Sense	GCACCGTCAAGGCTGAGAAC
Human GAPDH Antisense	TGGTGAAGACGCCAGTGGA
Rat MMP-1 Sense	GCTTAGCCTTCCTTTGCTGTTGC
Rat MMP-1 Antisense	GACGTCTTCACCCAAGTTGTAGTAG
Rat MMP-3 Sense	CGGTGGCTTCAGTACCTTTC
Rat MMP-3 Antisense	ACCTCCTCCCAGACCTTCA
Rat MMP-13 Sense	TGCATACGAGCATCCATCCC
Rat MMP-13 Antisense	CTCAAAGTGAACCGCAGCAC
Rat *β*-actin Sense	CACCCGCGAGTACAACCTTC
Rat *β*-actin Antisense	CCCATACCCACCATCACACC
NF*κ*B p65 siRNA Sense	GGCGAGAGGAGCACAGAUATT
NF*κ*B p65 siRNA Antisense	UAUCUGUGCUCCUCUCGCCTT
Negative control siRNA Sense	UUCUCCGAACGUGUCACGUTT
Negative control siRNA Antisense	ACGUGACACGUUCGGAGAATT

MMP, matrix metalloproteinase.

The article "Network Pharmacology-Based Strategy to Investigate the Mechanisms of Cibotium barometz in Treating Osteoarthritis" was published in 2022. Journal: Evid Based Complement Alternat Med.

**Table 2:** Chemical information of key components of *Cibotium barometz*.

No	RT (min)	Name	Formula	Ion	Cal. *m*/*z*	Mea. *m*/*z*	Error (ppm)	MS/MS
1	1.3	1,3,7-Trihydroxy-2-(3-methylbut-2-enyl)xanthone	C_18_H_16_O_5_	M-H	311.0924	311.0923	2.893	311.0923
2	2.9	Cochinchinol a	C_32_H_22_MgO_14_	M-H	653.0787	653.0798	3.651	315.05102
3	2.9	6-Deoxyjacareubin	C_18_H_14_O_5_	M + H	311.0914	311.0911	−0.965	311.0911
4	6.5	Cudraflavanone b	C_20_H_20_O_6_	M + H	357.1332	357.1337	1.219	357.1337
5	7.0	Naringenin	C_15_H_12_O_5_	M-H	271.0611	271.0615	5.165	151.0034, 107.0115
6	8.2	Kaempferol	C_15_H_10_O_6_	M-H	285.0404	285.04	0.636	285.04
7	8.3	Aspidinol	C_12_H_16_O_4_	M-H	223.0975	223.0971	2.755	223.0971
8	9.0	Cochinchinol b	C_30_H_18_CaO_14_	M-H	641.0249	641.0241	−2.84	301.035
9	22.4	Cudraxanthone q	C_23_H_22_O_5_	M-H	377.1394	377.1399	2.763	377.1399
10	24.0	Gerontoxanthone h	C_23_H_24_O_5_	M-H	379.155	379.1556	4.219	379.1556

## Data Availability

The data used to support the findings of this study are available from the corresponding author upon request.
